This article has been retracted.

# DEPDC1 promotes cell proliferation and suppresses sensitivity to chemotherapy in human hepatocellular carcinoma

**DOI:** 10.1042/BSR20190946

**Published:** 2019-07-10

**Authors:** Chao Zhou, Pu Wang, Mengtian Tu, Yi Huang, Fei Xiong, Yue Wu

**Affiliations:** 1 Department of Gastroenterology, Sichuan Academy of Medical Sciences and Sichuan Provincial People’s Hospital, Chengdu 610072, China; 2 Department of Laboratory Medicine, Sichuan Academy of Medical Sciences and Sichuan Provincial People’s Hospital, Chengdu 610072, China; 3 Department of Pharmacy, Sichuan Academy of Medical Sciences and Sichuan Provincial People’s Hospital, Chengdu 610072, China

**Keywords:** cell proliferation, chemotherapy resistance, DEPDC1, hepatocellular carcinoma, JNK signaling pathway

## Abstract

Background: Hepatocellular carcinoma (HCC) is one of the major causes of tumor-related morbidity and mortality worldwide. Accumulating evidence has revealed that aberrant expression of crucial cancer-related genes contributes to hepatocellular carcinogenesis. This study aimed to characterize the biological role of DEP domain containing 1 (DEPDC1), a novel cancer-related gene, in HCC and illuminate the potential molecular mechanisms involved.

Materials and methods: Quantitative real-time PCR (qRT-PCR), Western blotting and immunohistochemical (IHC) staining were used to characterize the expression patterns of DEPDC1 in tumorous tissues and adjacent normal tissues. Kaplan–Meier survival analysis was launched to evaluate the relationship between DEPDC1 expression and overall survival. CCK8 assay, colony formation and flow cytometry were performed to investigate the effects of DEPDC1 on HCC cell viability, clonogenic capability and cell apoptosis. Murine xenograft models were established to determine the effect of DEPDC1 on tumor growth *in vivo*. SP600125, a JNK specific inhibitor, was applied to carriy out mechanistic studies.

Results: DEPDC1 was significantly up-regulated in HCC tissues compared with para-cancerous tissues. Besides, patients with high DEPDC1 expression experienced a significantly shorter overall survival. Functional investigations demonstrated that DEPDC1 overexpression facilitated HCC cell proliferation and suppressed cell apoptosis, whereas DEPDC1 depletion inhibited cell proliferation and promoted cell apoptosis. Furthermore, DEPDC1 ablation suppressed tumorigenecity of HCC cells in murine xenograft models. Mechanistic studies uncovered that JNK signaling pathway mediated the promoting effects of DEPDC1 on HCC cell viability and chemotherapy resistance.

Conclusion: Collectively, our data may provide some evidence for DEPDC1 as a candidate therapeutic target for HCC.

## Background

Hepatocellular carcinoma, one of the most prevalent human malignancies, ranks the third most leading cause of tumor-related mortality worldwide, with approximately 600,000 deaths occurring annually [1–3]. It is estimated by American Cancer Research Society that more than 40,000 HCC cases were newly diagnosed and approximately 28,000 patients died of this cancer in the United States in 2017 [4]. It is widely acknowledged that drug resistance and distant metastasis are partially responsible for the high mortality of HCC patients [5–7]. Although significant progress has already been achieved in the diagnosis and treatment, the long-term prognosis is still rather poor. Hence, it is of great significance to develop novel and efficient therapeutic strategies. It is recognized that gene therapy may be a promising candidate therapy against HCC.

DEP domain containing 1 (DEPDC1), which is located at 1p31.3, is a highly conserved gene among many species ranging from *Caenorhabditis elegans* to human [8,9]. It is well documented that DEPDC1 encodes a highly conserved 92-kDa protein, which plays crucial roles in many biological processes, including cell proliferation, cell cycle progression, cell apoptosis and signaling transduction [10–12]. Recent studies have reported that DEPDC1 is implicated in diverse types of human cancers, such as bladder cancer [13], prostate cancer [14], nasopharyngeal carcinoma [15], lung adenocarcinoma [16] and glioma [17]. Nonetheless, the biological role of DEPDC1 in HCC remains largely unknown.

In the present study, we found that DEPDC1 was significantly up-regulated in HCC tissues compared with adjacent normal tissues. In addition, increased DEPDC1 expression was associated with poor prognosis of patients. Functional investigations demonstrated that DEPDC1 facilitated HCC cell proliferation and suppressed chemotherapy sensitivity. Furthermore, mechanistic studies revealed that c-Jun N-terminal kinase (JNK) signaling pathway mediated the oncogenic function of DEPDC1 in HCC. Collectively, this study may provide some evidence for DEPDC1 as a candidate therapeutic target against HCC.

## Materials and methods

### Patients and tissue samples

Tumor tissues and adjacent non-cancerous tissues were collected from 60 HCC patients who received surgical resection at Sichuan Academy of Medical Sciences and Sichuan Provincial People’s Hospital (Chengdu, China) between April 2010 and November 2016. Clinicopathological parameters of HCC patients were listed in Table 1. Overall survival time was defined as the interval between the date of primary surgery treatment and the date of death or last follow-up. All the patients gave their written consents. The present study was approved by the Ethics Committee of Xi’an Jiaotong University (Xi’an, China).

**Table 1:** Relationship between DEPDC1 mRNA expression and clinicopathological characteristics of HCC patients

Parameters	Number of cases	DEPDC1 expression		*P*-value
		High (*n* = 33)	Low (*n* = 27)	
Age				
<60	31	15	16	0.287
≧60	29	18	11	
Gender				
Female	28	16	12	0.755
Male	32	17	15	
Liver cirrhosis				
Yes	30	15	15	0.436
No	30	18	12	
Tumor size (cm)				
<5	26	9	17	0.006
≧5	34	24	10	
HBV infection				
Yes	28	18	10	0.176
No	32	15	17	
Lymph node metastasis				
Yes	33	17	16	0.549
No	27	16	11	
TNM stage				
I, II	26	10	16	0.024
III, IV	34	23	11	

### Cell lines and cell culture

Four human HCC cell lines (HepG2, SK-Hep1, Huh7 and Huh6) and normal human liver L02 cell line were purchased from Chinese Academy of Sciences (Shanghai, China). All the cells were cultured in DMEM medium (Gibco, Grand Island, NY, U.S.A.) containing 10% fetal bovine serum (FBS) in 5% CO_2_ humidified atmosphere at 37°C.

### Cell transfection

Cell transfection was performed using Lipofectamine 2000 according to the manufacturer’s protocols (Invitrogen, Carlsbad, CA, U.S.A.). DEPDC1 overexpression and knockdown studies were conducted using pcDNA3.1 and pLKO.1 (GenePharma Co. Ltd., Suzhou, China), respectively. Short hair RNA (shRNA) specially targeting DEPDC1 was designed by GenePharma and its sequence was as followed: 5′-GAACTATCAAGAGTAGTTCGT-3′. Transfection efficiency was examined after 48-h incubation.

### Quantitative real-time polymerase chain reaction (qRT-PCR)

Total RNA was extracted using RNeasy Kit (Qiagen, Valencia, CA) following the manufacture’s protocol. cDNA was synthesized by PrimeScript RT Master Mix (Takara, Dalian, China) based on the manufacturer’s instructions. The qRT-PCR analysis was carried out under an ABI Prism 7500 Fast Real-time PCR system using a SYBR Premix Ex Taq (Takara). GAPDH was used as an internal control. The sequences of primers were as followed: DEPDC1, forward 5′-ACGAAGGTATCCAGAATTG-3′and reverse 5′-AGATAATACCCAGTGAGGGA-3′; GAPDH, forward 5′-CTCCTCCACCTTTTGACGCTG-3′and reverse 5′-TCCTCTTGTGCTCTTGCTGG-3′. Relative DEPDC1 expression levels were calculated using 2^−△△*C*^_t_ method.

### Cell viability assays

Cell viability was measured using cell counting kit-8 (CCK8; Dojindo, Kumamoto, Japan). Cells (∼1 × 10^3^ per well) were seeded into 96-well plates and incubated for different time periods. Afterwards, 11 μl of CCK8 was added and incubated for another 4 h. The absorbance was determined using microplate reader (BioRad, Hercules, CA, U.S.A.) at 450 nm. The chemoresistance of HCC cells to cisplatin was examined by CCK8. Various concentrations of cisplatin were supplemented into 96-well plate and incubated for 12 h. Then, CCK8 was added and incubated for another 4 h. The absorbance was measured to evaluate the chemoresistance to cisplatin. All the experiments were conducted in triplicates.

### Colony formation assays

Colony formation assays were conducted to evaluate clonogenic capabilities of HCC cells. In brief, cells (∼1 × 10^3^ cells) were plated into six-well plates. The cells were cultured for 14 days to form colonies. Then the colonies were fixed by 4% paraformaldehyde for 20 min, followed by being stained with 0.2% Crystal Violet. Visible colonies were then photographed and counted under an invert light microscope (Nikon, Tokyo, Japan).

### Western blotting assays

Cell protein was extracted using RIPA lysis buffer (Takara) containing 1 nM PMSF (Invitrogen, Carlsbad, CA, U.S.A.) according to the manufacturer’s instructions. Then, 20 μg protein per well was electrophoresed in 10% SDS-PAGE gels and transferred onto PVDF membrane (Millipore, Bedford, MA, U.S.A.) and incubated with different primary antibodies, including anti-DEPDC1 (ab197246), anti-GAPDH (ab181603), anti-JNK (ab176645) and anti-p-JNK (ab107407) at 4°C overnight. The membrane was then incubated with HRP-labeled secondary at temperature for 2 h. The bands were detected using an ECL Western blotting kit (Invitrogen) and analyzed on a Gel Doc XR System (Bio-Rad Laboratories, Hercules, CA, U.S.A.).

### Cell apoptosis assays

Cell apoptosis was evaluated using Annexin-V FITC/PI Apoptosis Detection Kit (BD Bioscience, CA, U.S.A.) according to the manufacturer’s protocol. Cells were collected by low-speed centrifugation and rinsed twice with ice-cold PBS. Subsequently, cells were incubated with 300 μl of binding buffer. Afterward, cells were treated with 5 μl of PI and 5 μl of Annexin V-FITC (Invitrogen) at 4°C for 20 min in the dark. Then, cell apoptosis was detected by flow cytometry (Becton Dickinson).

### Murine Xenograft models

This animal protocol was approved by Animal Care and Use Committee of Sichuan Academy of Medical Sciences and Sichuan Provincial People’s Hospital (Chengdu, China). Ten 4-week-old male nude mice were purchased from the Model Animal Research Institute of Nanjing University (Nanjing, China). Xenograft models were established to evaluate the effects of DEPDC1 depletion on tumor growth *in vivo*. Briefly, Huh6 cells (5 × 10^6^) treated with pLKO.1 and pLKO.1-DEPDC1 were subcutaneously injected into the flanks of the mice. Tumor size was measured using slide caliper every 3 days, and tumor volumes were calculated according to the formula:volume (mm^3^) = [width^2^ (mm^2^) × length (mm)]/2. At day 21 post-inoculation, all the nude mice were killed, and the tumors were harvested and weighted.

### Immunohistochemistry (IHC)

Paraffin-embedded tissues were sectioned at 4.5-μm thickness. After being dewaxed and hydrated, sections were incubated with 3% H_2_O_2_ for 30 min to block the endogenous peroxidase (POD) activity. Following antigen recovery by repeated cooling and heating, 5% bovine serum albumin (BSA) was applied to block non-specific binding. The sections were then incubated with primary antibodies overnight at 4°C. Anti-DEPDC1 (ab197246) and anti-Ki67 (ab92742) were purchased from Abcam and used at a dilution of 1:500. After being rinsed with PBS three times for 5 min each, slices were treated with biotinylated secondary antibody for 1 h, followed by incubation with streptavidin-horseradish peroxidase (HRP) for 20 min. Diaminobenzidine substrate was used to visualize ZNF322-positive cells. Slides were then observed under a microscope (Nikon).

### Terminal deoxynucleotidyl transferase-mediated nick end labeling (TUNEL) assay

TUNEL analysis was conducted to monitor the apoptosis in the collected tumors using the In Situ Cell Death Detection Kit (Roche Diagnostic, Basel, Switzerland) following the manufacturer’s instructions. In brief, sample slides were incubated with 50 μl of TUNEL reaction mixture for 1 h at 37°C in the dark. After being rinsed with PBS three times, cells were then labeled with TdT labeling reaction mix. Positively stained cells were subsequently observed and photographed under an EVOS FL microscope (Thermo Fisher Scientific, Waltham, MA, U.S.A.).

### Statistical analysis

All the values were expressed as mean ± SD. SPSS18.0 software was applied to conduct statistical analysis. Differences between three or more groups were compared using analysis of variance (ANOVA) followed by Dunnett’s multiple comparison. Differences between two groups were compared using Student’s *t* test. The log-rank and Kaplan–Meier survival analysis were used to determine the correlation between DEPDC1 expression and overall survival. Fisher’s exact test was performed to evaluate the relationship between DEPDC1 expression and clinicopathological characteristics of patients. *P* < 0.05 was considered statistically significant.

## Results

### Increased expression of DEPDC1 predicts poor prognosis of HCC patients

Even though DEPDC1 has been identified as a crucial regulator in multiple types of human neoplasms, its role in HCC remains poorly understood. To characterize the biological role of DEPDC1 in HCC, we first determined its mRNA expression levels in 60 pairs of tumorous tissues and adjacent normal liver tissues by qRT-PCR analysis. As presented in Figure 1A, HCC tissues exhibited higher DEPDC1 mRNA expression levels than matched para-cancerous tissues. Besides, Western blotting analysis and IHC staining showed that DEPDC1 protein expression was significantly up-regulated in cancerous tissues compared with corresponding normal tissues (Figure 1B and C). To assess the relationship between DEPDC1 expression and overall survival of HCC patients, tumorous tissues were classified into high DEPDC1 expression group and low DEPDC1 expression group based on the average value of its mRNA expression levels. The log-rank test and Kaplan–Meier survival analysis demonstrated that patients with high DEPDC1 expression experienced a significantly shorter overall survival (Figure 1D). Furthermore, Fisher’s exact test showed that high DEPD1 expression was associated with larger tumor size and advanced TNM stage (Table 1). Consistently, we found that DEPDC1 was significantly up-regulated in HCC cell lines (HepG2, Huh7, SK-Hep1 and Huh6) in comparison with normal human liver L02 cells (Figure 1E). Collectively, our data indicate that increased DEPDC1 expression correlates with poor prognosis of HCC patients.

**Figure 1:** Increased expression of DEPDC1 predicts poor prognosis of HCC patients (**A**) DEPDC1 mRNA expression levels in 60 pairs of HCC tissues and adjacent non-cancerous tissues were examined by qRT-PCR analysis. (**B**) DEPDC1 protein expression levels in HCC tissues and matched normal tissues were detected by Western blotting analysis. (**C**) DEPDC1 protein expression in tumorous tissues and corresponding para-cancerous tissues were visualized by IHC. (**D**) HCC tissues were classified into high DEPDC1 expression group and low DEPDC1 expression group based on its mRNA expression levels. (**E**) DEPDC1 mRNA expression levels in normal human liver L02 cells and four HCC cell lines (HepG2, SK-Hep1, Huh7 and Huh6) were determined by qRT-PCR analysis; **P < 0.01; DEPDC1, DEP domain containing 1; HCC, hepatocellular carcinoma; qRT-PCR, quantitative real-time polymerase chain reaction; IHC, immunohistochemistry.

### DEPDC1 facilitates HCC cell proliferation and survival

In view of the findings mentioned above, we speculated that DEPDC1 was involved in human hepatocellular carcinogenesis and progression. To further investigate the biological role of DEPDC1 in HCC, we performed overexpression and knockdown studies in HepG2 cells (lowest endogenous DEPDC1 expression) and Huh6 cells (highest endogenous DEPDC1 expression), respectively. Transfection efficiency was determined by Western blotting (Figure 2A). As evident from CCK8 assays, DEPDC1 overexpression promoted Hep2G cell viability compared with control group, whereas DEPDC1 ablation inhibited Huh6 cell viability (Figure 2B). As shown in Figure 2C, DEPDC1 overexpression enhanced clonogenic ability of HepG2 cells in comparison with control group, while DEPDC1 depletion suppressed clonogenic capability of Huh6 cells. As displayed in Figure 2D, DEPDC1 overexpression repressed HepG2 cell apoptosis compared with control group, whereas DEPDC1 knockdown accelerated Huh6 cell apoptosis. Taken together, these results suggest that DEPDC1 promotes HCC cell proliferation and survival.

**Figure 2:** DEPDC1 facilitates HCC cell proliferation and survival (**A**) Transfection efficiency was evaluated by Western blotting assays after transfection with DEPDC1 expression vector or shRNA-DEPDC1. (**B**) Cell viability was measured by CCK8 assays after transfection with DEPDC1 expression vector or shRNA-DEPDC1. (**C**) Clonogenic ability was detected by colony formation assays after transfection with DEPDC1 expression vector or shRNA-DEPDC1. (**D**) Cell apoptosis was evaluated by flow cytometry after transfection with DEPDC1 expression vector or shRNA-DEPDC1; **P < 0.01; DEPDC1, DEP domain containing 1; HCC, hepatocellular carcinoma; shRNA, short hairpin RNA.

### DEPDC1 ablation suppresses tumorigenicity of HCC cells in murine xenograft models

To validate the effects of DEPDC1 *in vivo*, we established murine xenograft models by subcutaneous injection of shRNA-DEPDC1-treated Huh6 cells in the flank. As shown in Figure 3A, DEPDC1 knockdown significantly inhibited tumor growth *in vivo*. Besides, IHC staining demonstrated that less Ki67-positive cells were observed in the tumors collected from the shRNA-DEPDC1 group compared with control group (Figure 3B). Furthermore, TUNEL analysis revealed that DEPDC1 knockdown promoted cell apoptosis in the tumor compared with negative control group (Figure 3C). To sum up, our results suggest that DEPDC1 depletion inhibits tumor growth *in vivo*.

**Figure 3:** DEPDC1 ablation suppresses tumorigenicity of HCC cells in murine xenograft models (**A**) shRNA-DEPDC1 treated Huh6 cells were subcutaneously injected into the flanks of the mice (*n* = 5). Tumor volume was measured by slide caliper every 3 days; the mice were killed and tumors were weighed at day 21 post-implantation. (**B**) Ki67 protein expression in the collected tumors were visualized by IHC staining. (**C**) Apoptotic cells in the harvested tumors were determined by TUNEL assays; **P < 0.01; DEPDC1, DEP domain containing 1; HCC, hepatocellular carcinoma; shRNA, short hairpin RNA; TUNEL, terminal deoxynucleotidyl mediated nick end labeling.

### DEPDC1 promotes activation of JNK signaling pathway in HCC cells

Previous studies have demonstrated that JNK signaling pathway plays critical roles in cancer cell proliferation, growth and motility. To clarify the potential molecular mechanisms underlying HCC, we evaluated the effects of DEPDC1 overexpression or ablation on JNK signaling pathway. As presented in Figure 4A, DEPDC1 overexpression promoted the phosphorylation of JNK compared with control group, whereas DEPDC1 knockdown suppressed the phosphorylation of JNK. Furthermore, Western blotting analysis showed that usage of SP600125, a specific JNK inhibitor, reversed the promoting effects of DEPDC1 overexpression on the phosphorylation of JNK (Figure 4B). Besides, we found that JNK specific inhibitor SP600125 also reversed the inhibitory effect of DEPDC1 overexpression on HepG2 cell apoptosis (Figure 4C). Taken together, these findings indicate that DEPDC1 promotes activation of JNK signaling pathway in HCC cells.

**Figure 4:** DEPDC1 promotes activation of JNK signaling pathway in HCC cells (**A**) JNK and p-JNK protein expression levels were examined by Western blotting in DEPDC1 overexpression group and DEPDC1 depletion group, respectively. (**B**) JNK and p-JNK protein expression levels were determined by Western blotting after usage of JNK specific inhibitor SP600125 in DEPDC1 overexpression group. (**C**) FCM analysis was performed to evaluate the effect of JNK specific inhibitor SP600125 on apoptosis of HepG2 cells overexpressing DEPDC1; **P<0.01; DEPDC1, DEP domain containing 1; JNK, c-Jun N-terminal kinase; HCC, hepatocellular carcinoma; p-JNK, phosphorylated c-Jun N-terminal kinase.

### DEPDC1 depletion enhances sensitivity of HCC cells to chemotherapy through JNK signaling pathway

To verify the potential molecular mechanisms by which DEPDC1 promotes HCC viability and survival, we performed subsequent studies. As displayed in Figure 5A, DEPDC1 overexpression enhanced viability of cisplatin-treated HepG2 cells compared with control group, whereas DEPDC1 depletion inhibited viability of cisplatin-treated Huh6 cells. Furthermore, FCM analysis demonstrated that DEPDC1 overexpression inhibited apoptosis of cisplatin-treated HepG2 cells, whereas DEPDC1 depletion promoted apoptosis of cisplatin-treated Huh6 cells (Figure 5B). Besides, we found that JNK specific inhibitor SP600125 suppressed viability and survival of cisplatin-treated Huh6 cells compared with control group, suggesting that SP600125 possesses similar effect on HCC cell viability and survival to DEPDC1 ablation (Figure 5C). Collectively, these results indicate that DEPDC1 ablation enhances sensitivity of HCC cells to chemotherapy through JNK pathway.

**Figure 5:** DEPDC1 depletion enhances sensitivity of HCC cells to chemotherapy through JNK signaling pathway (**A**) Cell viability was detected by CCK8 assay after treatment with different concentrations of cisplatin for 12 h. (**B**) Cell apoptosis was evaluated using flow cytometry after treatment with 10 μM cisplatin for 12 h. (**C**) Cell viability from DMSO group and SP600125 group was determined by CCK8 assays after treatment with various concentration of cisplatin for 12 h, respectively; cell apoptosis from DMSO and SP600125 group was examined by flow cytometry after treatment with 10 μM cisplatin for 12 h; **P < 0.01; DEPDC1, DEP domain containing 1; HCC, hepatocellular carcinoma; JNK, c-Jun N-terminal kinase.

## Discussion

HCC, one of the most lethal malignancies, has imposed great pressure on public health and posed enormous threats to human life worldwide [18,19]. It is widely acknowledged that dys-regulation of tumor-related signaling pathways is implicated in human carcinogenesis and development [20–24]. Furthermore, targeting dysregulated cancer-related signal pathways is considered as a promising therapeutic strategy for HCC patients. Even through great advances have already been achieved in the therapy of HCC, the long-term prognosis remains rather discouraging. Hence, novel and efficient therapeutic strategies are in urgent demand. Accumulating evidence has demonstrated that aberrant expression of crucial tumor-related genes contributes to tumorigenesis and malignant progression of human HCC. Wang et al. [25] demonstrated that FAM83D was up-regulated and promoted cell proliferation through activating MEK/ERK signaling pathway in HCC. Chen et al. [26] found that IQGAP1 was overexpressed and promoted cell proliferation by activating Akt signaling in HCC. Fang et al. [27] reported that FBI-1 promoted cell proliferation and enhanced chemotherapy resistance in HCC. Dai et al. [28] revealed that GOLPH3 promoted cell aggressiveness via activating NF-κB pathway in HCC. Despite the fact that a great deal of studies have focused on the ectopic expression of cancer-related genes up to now, much attention should be paid to identifying more genes which are implicated in the initiation and development of HCC.

Past studies showed that DEPDC1 was implicated in multiple types of human neoplasms. Harada and co-workers [13] demonstrated that DEPDC1 contributed to bladder cancer oncogenesis. Huang and co-workers [14] reported that DEPDC1 promoted prostate cancer cell proliferation and tumor growth via activation of E2F signaling pathway. Feng et al. [15] revealed that DEPDC1 facilitated nasopharyngeal carcinoma cell cycle progression and motility. Wang and co-workers [17] found that increased DEPDC1 expression was associated with poor prognosis of patients with lung adenocarcinoma. However, the biological role of DEPDC1 in HCC remains poorly understood. Hence, it may be worthy to characterize the role of DEPDC1 in HCC.

To investigate the role of DEPDC1 in HCC, we first analyzed the expression of DEPDC1 in tumorous tissues and matched adjacent non-cancerous tissues and found that DEPDC1 was highly expressed in HCC tissues. In addition, we noticed that increased DEPDC1 expression predicts poor prognosis of patients. Functional studies showed that DEPDC1 overexpression facilitated HCC cell proliferation, inhibited cell apoptosis and chemotherapy sensitivity, whereas DEPDC1 depletion suppressed cell proliferation, promoted cell apoptosis and chemotherapy sensitivity. Emerging evidence has demonstrated that abnormal control of cancer-related signaling transduction pathways contributes to HCC initiation and malignant development [29–31]. It is well documented that activation of JNK signaling pathway contributes to carcinogenesis and tumor progression of various types of human malignancies [32–35]. In the present study, mechanistic investigations identified that DEPDC1 overexpression promoted HCC cell viability and chemotherapy resistance by activating JNK signaling pathway, while DEPDC1 knocked suppressed cell viability and chemotherapy resistance by down-regulating JNK pathway; meanwhile, JNK specific inhibitor SP600125 was observed to have similar effects to DEPDC1 depletion, indicating that JNK pathway mediated the oncogenic effects of DEPDC1 in HCC. DEPDC1-induced JNK pathway activation may be attributed to its recruiting phosphorylases to facilitate phosphorylation of JNK1/2 proteins [36]. There is no doubt that some limitations exist in the current studies. In our further work, we will conduct corresponding studies to explore the effects of DEPDC1 on HCC cell motility and metastasis to better characterize its biological functions.

In conclusion, the present study for the first time demonstrated that DEPDC1 was significantly up-regulated in HCC tissues compared with matched non-cancerous tissues and that high DEPDC1 expression correlated with poor prognosis of patients. Furthermore, our findings indicate that DEPDC1 promotes HCC cell proliferation and suppresses chemotherapy sensitivity through activating JNK signaling pathway. Therefore, our study provides some new insights into understanding the molecular mechanisms underlying hepatocellular carcinogenesis, implying that DEPDC1 may be used as a promising candidate therapeutic target against HCC.

## Abbreviations

CCK8: cell counting kit-8
DEPDC1: DEP domain containg 1
HCC: hepatocellular carcinoma
IHC: immunohistochemical
JNK: c-Jun N-terminal kinase
